# Usefulness of the Atherosclerosis Risk Score for Patients With Acute Infarction in the Lenticulostriate Artery Region

**DOI:** 10.7759/cureus.23591

**Published:** 2022-03-28

**Authors:** Hikaru Nakamura, Kei Sato, Kosuke Hirayama, Yukishige Hayashi, Yoshiharu Tokunaga

**Affiliations:** 1 Neurosurgery, Nagasaki Prefecture Shimabara Hospital, Shimabara, JPN

**Keywords:** lenticulostriate artery, striatocapsular infarction, branch atheromatous disease, lacunar infarction, suita score, framingham risk score

## Abstract

Background and purpose

Internal carotid artery intima-media thickness (IMT) and pulse wave velocity (PWV) are risk factors of cerebrovascular disease and coronary artery disease. They are known as independent predictors of arteriosclerotic disease. It has been reported that IMT and PWV are useful factors for predicting stroke subtype and/or outcome.

Coronary artery disease onset is proportional to atherosclerosis progression, and the Framingham Risk Score (FRS) and Suita score (SS) are standard risk predictors. This study examined whether FRS and SS can be useful for patient outcomes with acute infarction in the lenticulostriate artery (LSA) region without special tests or invasive procedures while using IMT or PWV as predictive factors.

Methods

We screened 629 consecutive patients with ischemic stroke and reviewed 84 patients with acute infarction in the LSA region who were admitted between January 2018 and December 2020. An early deterioration (ED) group was defined. In addition, the clinical characteristics, FRS, SS, treatment therapy, and neurovascular findings were evaluated.

Results

FRS and SS (FRS: 11.6 vs. 8.3, *p *< 0.01, SS: 58.2 vs. 53.7, *p *= 0.01, respectively), pre-symptomatic modified Rankin Scale (mRS) (p = 0.03), mRS at discharge (p < 0.01), and deterioration of manual muscle test (MMT) (<0.01) were significantly higher in patients in the ED (34 patients) group than in the no-ED group (54 patients). FRS and SS were correlated with mRS deterioration (FRS: r = 0.47;* p *< 0.01, SS: r = 0.23; *p *= 0.03). Among the laboratory parameters, total cholesterol (TC) (p < 0.01) and low-density lipoprotein cholesterol (LDL-C) (p < 0.01) were significantly higher in the ED group, and no significant differences in any acute therapeutic interventions.

Conclusion

Atherosclerosis risk scores, such as FRS and SS, may be useful for predicting outcomes in patients with acute LSA-region infarctions within 48 hours of onset.

## Introduction

Ischemic stroke is one of the leading causes of death and severe disability. Thus, accurate diagnosis and early prediction of disease progression are essential to choose treatment interventions and use limited medical resources appropriately.

Previously, cerebral infarction was classified according to the diagnostic criteria of the Trial of ORG 10172 in acute stroke treatment [1]. However, patients with acute lenticulostriate artery (LSA) infarctions have several stroke subtypes, including lacunar infarction (LI), branch atheromatous disease (BAD), and striatocapsular infarction (SCI), and more complicated course than other penetrating arteries [2].

Recently, small subcortical infarctions caused by atherosclerosis have been reported as strong predictors for progressive motor deficits [3]. Internal carotid artery intima-media thickness (IMT) and pulse wave velocity (PWV) are predictors of cerebrovascular disease and coronary artery disease. They are known as independent predictors of arteriosclerotic disease. It has been reported that IMT and PWV are useful factors for predicting stroke subtype and/or outcome [4,5,6,7].

Although no specialized scoring system for evaluating atherosclerosis in stroke is currently known, the onset of coronary artery disease is proportional to the progression of atherosclerosis, and the Framingham risk score (FRS) or Suita score (SS) are standard risk predictors. FRS is a sex-specific algorithm used to estimate the 10-year cardiovascular risk of an individual that was first developed based on data obtained from the Framingham Heart Study of 1998 [8]. It has been used worldwide for a long time. However, the risk of developing myocardial infarction is extremely low in the Japanese population compared to that in the Western population. In addition, the risk of developing coronary artery disease is low in chronic kidney disease (CKD) patients; therefore, SS, developed in 2014 based on the Suita study, could evaluate such patients [9].

Several studies have examined factors predicting outcomes in patients with LSA-region infarctions based on clinical features, imaging findings, or specific laboratory data. However, in this study, using two arteriosclerosis risk scores (FRS and SS), we examined the possibility of easily predicting outcomes in patients with acute infarction in the LSA region while using IMT or PWV as predictive factors, and without special imaging or invasive examinations.

## Materials and methods

Participants

Approval for this study and a waiver of informed consent were obtained from the Institutional Review Board of Nagasaki Prefecture Shimabara Hospital because of its retrospective nature.

We screened 629 consecutive patients with ischemic stroke and reviewed 84 patients between January 2018 and December 2020 within 48 hours of the onset of acute infarction in the LSA region (Figure 1). The early deterioration (ED) group was defined by worsening of the pre-symptomatic modified Ranking Scale (mRS) by two or more stages at discharge, and the remaining patients were categorized into the no-early deterioration (no-ED) group. We compared these two groups, and mRS deterioration was defined as the difference between pre-symptomatic mRS and mRS at discharge.

**Figure 1:** Flowchart of patient selection. LSA: Lenticulostriate artery.

FRS was calculated based on age, sex, total cholesterol (TC), triglyceride (TG), low-density lipoprotein cholesterol (LDL-C), high-density lipoprotein cholesterol (HDL-C), systolic and diastolic blood pressure, diabetes, and current smoking status [8]. In addition, the SS LDL-C version was calculated based on age, HDL-C, LDL-C, systolic blood pressure, diabetes mellitus, current smoking status, and estimated glomerular filtration rate (eGFR) [9].

Acute infarction was defined by neurological deficits, such as pure motor hemiparesis and sensory-motor stroke, within 48 hours from the onset of a corresponding hyperintense lesion on MRI with diffusion-weighted imaging (DWI) and hypo-intense lesion on an apparent diffusion coefficient map.

Table 1 shows the clinical characteristics evaluated on admission and the following information collected from medical records: age (years); sex; time from onset to admission (hours); FRS; SS; manual muscle test (MMT) deterioration from the time of admission to discharge; vascular risk factors, such as hypertension, diabetes mellitus, hyperlipidemia, eGFR, current smoking status, atrial fibrillation, family history of ischemic stroke and blood pressure; National Institutes of Health Stroke Scale scores (NIHSS); pre-symptomatic mRS; and mRS at discharge. Laboratory parameters were obtained from routine blood examination, including TC, TG, LDL-C, and HDL-C. Tissue plasminogen activator (tPA), single-antiplatelet therapy (SAPT), double-antiplatelet therapy (DAPT), statin, anticoagulant, argatroban, ozagrel, and edaravone were administered after admission.

**Table 1:** Baseline characteristics of the study population. no-ED: No early deterioration group; ED: Early deterioration group; MMT: Manual muscle test; eGFR: Estimated glomerular filtration rate; NIHSS: National Institutes of Health Stroke Scale; mRS: modified Ranking Scale; TC: Total cholesterol; TG: Triglyceride; LDL-C: Low-density lipoprotein cholesterol; HDL-C: High-density lipoprotein cholesterol; tPA: Tissue plasminogen activator; SAPT: Single antiplatelet therapy; DAPT: Double antiplatelet therapy.

	no-ED group (n = 50)	ED group (n = 34)	p-value
Age (years)	73.1 (±13.4)	76.5 (±11.8)	0.23
Male sex (%)	30 (60%)	18 (52.9%)	0.65
Time to admission (hours)	12.7 (±12.9)	13.9 (±13.8)	0.69
Framingham risk score	8.32 (±3.7)	11.6 (±3.3)	<0.01
Suita score	53.7 (±7.6)	58.2 (±8.6)	0.01
Deterioration of MMT	17 (34%)	17 (50%)	<0.01
Risk factors			
・Hypertension	39 (78%)	22 (64.7%)	0.22
・Diabetes Mellitus	11 (22%)	10 (29.4%)	0.45
・Hyperlipidemia	14 (28%)	7 (20.6%)	0.61
・eGFR	60.8 (±15.1)	60.4 (±19.5)	0.91
・Current smoking	8 (16%)	9 (26.5%)	0.28
・Atrial fibrillation	8 (16%)	3 (8.8%)	0.51
・Family history of ischemic stroke	9 (18%)	1 (2.9%)	0.04
Systolic blood pressure (mmHg)	161.5 (±22.3)	166.5 (±31.7)	0.4
Diastolic blood pressure (mmHg)	92.7 (±18.4)	92.9 (±17.7)	0.95
NIHSS score on admission	4 (±6.0)	3.3 (±3.1)	0.53
Pre-symptomatic mRS	1.12 (±1.5)	0.5 (±0.79)	0.03
mRS at discharge	1.6 (±1.4)	3.2 (±1.1)	<0.01
Laboratory parameters			
・TC	193.5 (±41.5)	221.5 (±45.2)	<0.01
・TG	123 (±70.7)	128.4(±53.7)	0.71
・LDL-C	111.7 (±33.3)	134.7 (±37.2)	<0.01
・HDL-C	57.7 (±17.4)	58.4 (±17.9)	0.86
Treatment			
・tPA	8 (16%)	2 (5.9%)	0.19
・SAPT	24 (48%)	14 (41.2%)	0.66
・DAPT	18 (36%)	18 (52.9%)	0.18
・Statin	14 (28%)	11 (32.4%)	0.81
・Anticoagulant	8 (16%)	3 (8.8%)	0.51
・Argatroban	30 (60%)	23 (67.6%)	0.5
・Ozagurel	7 (14%)	4 (11.8%)	1
・Edaravone	32 (64%)	21 (61.8%)	1

Neurovascular imaging

MRI was performed using a 1.5-Tesla Siemens MRI scanner (Siemens Avanto; Siemens, Erlangen, Germany) or 3.0-Tesla Siemens MRI scanner (Siemens Skyra; Siemens, Erlangen, Germany). Axial DWI was obtained using spin-echo echo-planar sequences with 5-mm-thick slices and 1-mm inter-slice gaps. The horizontal and vertical infarct size was measured as the maximal diameter of the lesion, and the infarct slice number used to evaluate the vertical extension of the lesion was defined as the number of infarcts visible on DWI.

LI was defined as a cerebral infarction with a lateral diameter of less than 15 mm and less than three slices in the perforator region, BAD as an infarction that did not correspond to LI in the LSA region and spanned more than three slices in horizontal slice, and SCI as a subcortical infarction with a maximum diameter of 20 mm or more, including the Heubner artery or anterior choroidal artery region in several cases in the LSA region.

Magnetic resonance angiography (MRA) was performed to identify severe stenosis or occlusion in the clinically relevant artery, the internal carotid artery (ICA), and the M1 portion of the middle cerebral artery (MCA) from which most of the LSAs branch. Severe stenosis was defined as a single reduction of more than 70% of the nearest normal-sized vessel or focal signal loss. All image analyses were performed by experienced neurologists blinded to all clinical data.

Statistical analysis

In the univariate analyses, variables between the two groups were compared using Student’s t-test for continuous variables and Chi-squared test for categorical variables as appropriate. Correlation between atherosclerosis risk scores and mRS deterioration was examined using Spearman’s rank-order correlation coefficient. Multivariate logistic regression analyses were not performed due to the small number of patients. All statistical analyses were considered statistically significant with p < 0.05. All statistical analyses were performed using EZR, a modified version of the R commander designed to add statistical functions frequently used in biostatistics [10].

## Results

Figure 1 shows that we screened 629 consecutive patients with ischemic stroke and excluded 540 patients. Finally, 84 patients were included. The clinical characteristics and laboratory parameters compared between the two groups are presented in Table 1. A total of 84 consecutive patients with acute LSA region infarctions were admitted to our hospital during the study period.

FRS (p < 0.01), SS (p = 0.01), pre-symptomatic mRS (p = 0.03), mRS at discharge (p < 0.01), and deterioration of MMT (<0.01) were significantly higher in patients in the ED group than in the no-ED group. No significant differences in age (years), sex, time to admission (hours), systolic and diastolic blood pressure, NIHSS score on admission, and vascular risk factors, such as hypertension, diabetes mellitus, hyperlipidemia, current smoking status, and eGFR, were observed between the two groups. Moreover, the family history of ischemic was significantly higher in the no-ED group (p = 0.04).

Among the laboratory parameters, TC (p < 0.01) and LDL-C (p < 0.01) were significantly higher in the ED group than in the no-ED group, and no significant differences in TG and HDL-C were noted. For acute therapeutic interventions, the use of tPA, SAPT, DAPT, statin, anticoagulant, argatroban, ozagrel, and edaravone were compared between the two groups. However, no significant differences were observed between them.

The MRI and MRA characteristics were compared, and the results are shown in Table 2. As a stroke subtype, the incidence of LI, BAD, and SCI was not significantly different between the two groups. However, the stroke location of right (no-ED, 61.8% vs. ED, 38%, p = 0.045) and severe stenosis (no-ED, 32.4% vs. ED, 12%, p = 0.03) were significantly higher in the ED group than in the no-ED group. On admission, vertical (no-ED 12.5±5.5 mm vs. ED, 15.4±6.1 mm; p = 0.02) sizes on DWI were significantly different; however, no significant difference was found in the horizontal size. Upon follow-up, the horizontal (no-ED, 11.3±4.9 mm vs. ED, 17.3±7.0 mm; p < 0.01) and vertical (no-ED, 14.8±5.5 mm vs. ED, 18.8±7.1 mm; p < 0.01) sizes on DWI were both significantly different.

**Table 2:** MRI characteristics in the no-ED and ED groups. no-ED: No early deterioration group; ED: Early deterioration group; LI: Lacunar infarction; BAD: Branch atheromatous disease; SCI: Striatocapsular infarction; DWI: Diffusion-weighted imaging.

	no-ED group (n = 50)	ED group (n = 34)	p-value
Stroke subtype			
・LI	28 (56%)	11 (32.4%)	0.07
・BAD	18 (36%)	17 (50%)	0.26
・SCI	4 (8%)	6 (17.6%)	0.3
Right, location	19 (38%)	21 (61.8%)	0.045
Severe stenosis	6 (12%)	11 (32.4%)	0.03
DWI findings on admission			
・Horizontal size (mm)	11.03 (±7.76)	13.044 (±5.7)	0.2
・Vertical size (mm)	12.5 (±5.5)	15.4 (±6.1)	0.02
DWI findings on follow-up			
・Horizontal size (mm)	11.3 (±4.9)	17.3 (±7.0)	<0.01
・Vertical size (mm)	14.8 (±5.5)	18.8 (±7.1)	<0.01

As Figure 2 shows, there was a significant positive correlation between FRS or SS and mRS deterioration (FRS: r = 0.47; p < 0.01, SS: r = 0.23; p = 0.03).

**Figure 2:** Correlation between atherosclerosis risk score and mRS deterioration from pre-symptomatic stage to discharge. (A) There was a significant correlation between FRS and mRS deterioration from pre-symptomatic ｍRS to discharge (r = 0.47, p < 0.01). (B) There was a significant correlation between SS and mRS deterioration from pre-symptomatic ｍRS to discharge (r = 0.23, p = 0.03).

## Discussion

This is the first study showing the usefulness of atherosclerosis risk scores, such as FRS or SS, at predicting outcomes in patients with acute infarctions in the LSA region.

Patients with acute LSA region infarctions have various types of subcortical infarcts, including LI, BAD, and SCI. LI is a single-penetrating-branch infarction and is defined as an infarction caused by lesions of the penetrating branch itself, such as lipohyalinosis or microatheroma [11,12]. BAD is defined as an occlusion in the vicinity of the bifurcation of a penetrating branch from the mother artery by atheroma plaque [2,13]. SCI is a clinical subtype of subcortical infarction in the entirety or part of the LSA region. The cause is atherosclerotic changes in the major cerebral artery, and cardiogenic cerebral embolism accounts for the majority of cases [14-17]. Symptoms mostly worsen atherosclerosis-derived BAD or SCI.

Previous studies showed that carotid artery IMT, known as a risk factor for cerebrovascular disease and coronary artery disease and an independent predictor of atherosclerotic disease, can predict LI or distinguish other stroke subtypes from LI [5,7]. An association between PWV and outcomes in patients with cerebral infarction has also been reported [6]. In the present study, we did not show a significant difference of FRS and SS in LI patients from other stroke subtypes (FRS: LI, 9.49±3.97 vs. BAD, 9.71±3.97, p = 0.81; SS: LI, 56.7±8.31 vs. BAD, 54.8±8.82, p = 0.36; FRS: LI, 9.49±3.97 vs. SCI, 9.7±3.1, p = 0.88; and SS: LI, 56.7±8.31 vs. SCI. 53.9±5.95, p = 0.33), and LI tended to be higher in no-ED, but no significant difference was shown (Table 2).

Moreover, as shown in Figure 2, we also found a significant correlation between atherosclerosis risk score and mRS deterioration from pre-symptomatic ｍRS at discharge.

Based on these results, the atherosclerosis risk score may be useful for predicting outcomes for patients with acute infarction in the LSA region, similar to other atherosclerosis indicators. As shown in Table 1, the ratio of MMT degradation was significantly high in the ED group. Thus it is possible that neurological deterioration was the cause of ED. However, neither FRS nor SS showed a significant difference in the stroke subtypes, and it is speculated that there are cases where the outcome is poor, even if the infarct size is small.

For this reason, we consider the neurological adverse effects of atherosclerosis and the effects of arteriosclerosis on other poor outcome factors. As a neurological adverse effect of atherosclerosis, decreased protective factors, such as nitric oxide (NO), endogenous tPA, decreased collateral circulation, atherosclerotic cerebral microcirculatory disorders, and gradual obstruction of penetrating branches, may cause damage to the vascular endothelium and blood-brain barrier (BBB), resulting in damage to the brain parenchyma [18-24]. In addition, pulsatility of LSA and blood flow from MCA to LSA decrease with increasing cerebral vascular resistance [25]. In patients with acute ischemic stroke, it has been reported that elderly patients and patients with diabetes or hypertension have poor collateral circulation. Therefore, we speculate that patients with high atherosclerosis risk scores may also have low ischemic tolerance in the LSA area [26]. For these reasons, atherosclerosis risks may have a negative effect on neurological outcomes.

Patients with a high atherosclerosis risk score may have advanced atherosclerosis. Their general condition is poorer than patients with a low score. It is said that the complication rate of pneumonia and urinary tract infection, which are complications in the acute stage of stroke, is high for older people and smokers, which are both atherosclerosis risk factors [27-30]. Additionally, predisposition to arteriosclerosis, such as hypertension, dyslipidemia, and diabetes, is known as a risk factor for the development of dementia, which is an inhibitor of stroke rehabilitation [31]. Thus, effective rehabilitation may be inhibited in patients with a high arteriosclerosis risk score.

As shown by the study results, the assessment of atherosclerosis risk at the time of admission may be beneficial in predicting outcomes. However, appropriate therapeutic intervention is required to prevent the worsening of neurological symptoms from the early stage. As Table 1 shows, we evaluated several treatments and found that tPA infusion tended to be higher in the no-ED group; however, no significant difference was shown. There was also no significant difference in the use of antiplatelet agents, statin, argatroban, ozagrel, edaravone, and the presence of cardiogenic cerebral embolism and the use of anticoagulants. Therefore, further investigation is necessary.

This study is limited by its retrospective nature and the small number of recruited patients. Hence, further prospective studies with larger numbers of patients are warranted to confirm these results.

## Conclusions

In addition to the neurological adverse effects of atherosclerosis, patients with a high atherosclerosis risk score may have a poorer condition than patients with a low score, and the complication rate of pneumonia, urinary tract infection, or dementia may be high. Thus, atherosclerosis risk scores, such as FRS and SS, may be useful for predicting outcomes in patients with acute LSA-region infarctions within 48 hours of onset. Additionally, if an effective treatment can be established, it may also be useful in initiating appropriate therapeutic interventions without special tests or invasive procedures.

## References

[1] Ay H, Furie KL, Singhal A, Smith WS, Sorensen AG, Koroshetz WJ (2005). An evidence-based causative classification system for acute ischemic stroke. Ann Neurol.

[2] Marinkovic SV, Milisavljevic MM, Kovacevic MS, Stevic ZD (1985). Perforating branches of the middle cerebral artery. Microanatomy and clinical significance of their intracerebral segments. Stroke.

[3] Hallevi H, Chernyshev OY, El Khoury R, Soileau MJ, Walker KC, Grotta JC, Savitz SI (2012). Intracranial atherosclerosis is associated with progression of neurological deficit in subcortical stroke. Cerebrovasc Dis.

[4] Duan S, Zhang S, Li L, Ren C, Xie J (2017). Carotid artery intima-media thickness associated with prognosis of intracranial branch atheromatous disease. Int J Neurosci.

[5] Cupini LM, Pasqualetti P, Diomedi M (2002). Carotid artery intima-media thickness and lacunar versus nonlacunar infarcts. Stroke.

[6] Saji N, Kimura K, Kawarai T, Shimizu H, Kita Y (2012). Arterial stiffness and progressive neurological deficit in patients with acute deep subcortical infarction. Stroke.

[7] Kokubo Y, Watanabe M, Higashiyama A, Nakao YM, Nakamura F, Miyamoto Y (2018). Impact of intima-media thickness progression in the common carotid arteries on the risk of incident cardiovascular disease in the Suita study. J Am Heart Assoc.

[8] Wilson PW, D'Agostino RB, Levy D, Belanger AM, Silbershatz H, Kannel WB (1998). Prediction of coronary heart disease using risk factor categories. Circulation.

[9] Nishimura K, Okamura T, Watanabe M (2014). Predicting coronary heart disease using risk factor categories for a Japanese urban population, and comparison with the framingham risk score: the Suita study. J Atheroscler Thromb.

[10] Kanda Y (2013). Investigation of the freely available easy-to-use software 'EZR' for medical statistics. Bone Marrow Transplant.

[11] Yamamoto Y, Ohara T, Hamanaka M, Hosomi A, Tamura A, Akiguchi I (2011). Characteristics of intracranial branch atheromatous disease and its association with progressive motor deficits. J Neurol Sci.

[12] Miller FC (1991). Lacunar infarcts - A review. Cerebrovasc Dis.

[13] Caplan LR (2015). Lacunar infarction and small vessel disease: pathology and pathophysiology. J Stroke.

[14] Bladin PF, Berkovic SF (1984). Striatocapsular infarction: large infarcts in the lenticulostriate arterial territory. Neurology.

[15] Donnan GA, Bladin PF, Berkovic SF, Longley WA, Saling MM (1991). The stroke syndrome of striatocapsular infarction. Brain.

[16] Weiller C, Ringelstein EB, Reiche W, Thron A, Buell U (1990). The large striatocapsular infarct. A clinical and pathophysiological entity. Arch Neurol.

[17] Nicolai A, Lazzarino LG, Biasutti E (1996). Large striatocapsular infarcts: clinical features and risk factors. J Neurol.

[18] Castillo J (1999). Deteriorating stroke: diagnostic criteria, predictors, mechanisms and treatment. Cerebrovasc Dis.

[19] Asahi M, Huang Z, Thomas S (2005). Protective effects of statins involving both eNOS and tPA in focal cerebral ischemia. J Cereb Blood Flow Metab.

[20] Nakamura K, Saku Y, Ibayashi S, Fujishima M (1999). Progressive motor deficits in lacunar infarction. Neurology.

[21] Steinke W, Ley SC (2002). Lacunar stroke is the major cause of progressive motor deficits. Stroke.

[22] Kim J, Cha MJ, Lee DH (2011). The association between cerebral atherosclerosis and arterial stiffness in acute ischemic stroke. Atherosclerosis.

[23] Gasecki D, Rojek A, Kwarciany M (2012). Aortic stiffness predicts functional outcome in patients after ischemic stroke. Stroke.

[24] Wardlaw JM (2010). Blood-brain barrier and cerebral small vessel disease. J Neurol Sci.

[25] Schnerr RS, Jansen JF, Uludag K, Hofman PA, Wildberger JE, van Oostenbrugge RJ, Backes WH (2017). Pulsatility of lenticulostriate arteries assessed by 7 Tesla flow MRI-measurement, reproducibility, and applicability to aging effect. Front Physiol.

[26] Wiegers EJ, Mulder MJ, Jansen IG (2020). Clinical and imaging determinants of collateral status in patients with acute ischemic stroke in MR CLEAN trial and registry. Stroke.

[27] Langhorne P, Stott DJ, Robertson L (2000). Medical complications after stroke: a multicenter study. Stroke.

[28] Langdon PC, Lee AH, Binns CW (2009). High incidence of respiratory infections in 'nil by mouth' tube-fed acute ischemic stroke patients. Neuroepidemiology.

[29] Hoffmann S, Malzahn U, Harms H (2012). Development of a clinical score (A2DS2) to predict pneumonia in acute ischemic stroke. Stroke.

[30] Ivan CS, Seshadri S, Beiser A, Au R, Kase CS, Kelly-Hayes M, Wolf PA (2004). Dementia after stroke: the Framingham Study. Stroke.

[31] Popović IM, Serić V, Demarin V (2007). Mild cognitive impairment in symptomatic and asymptomatic cerebrovascular disease. J Neurol Sci.

